# MRNA Profiling Involved in Triggering of STAT1 with Regulatory Involvement of IRF7, PTPRF, and miR-145p in Patients Suffering from Gall Bladder Carcinoma

**DOI:** 10.1155/2022/1770643

**Published:** 2022-01-07

**Authors:** Weiwei Zhao, Yanxuan Gong, Yugang Chen

**Affiliations:** ^1^Three Department of General Surgery (Oncology Surgery), The Second People's Hospital in Lanzhou, Lanzhou, China; ^2^Xi'an International University, Xi'an, China

## Abstract

**Background:**

Gall Bladder Cancer (GBC) is a type of extremely malignant tumor, which has high incidences of mortality. There is rare information about its mechanisms of invasion and gene expression regulations. microRNA-155 (miR-155) has mostly been reported to be over expressed in cases of solid tumors and hematopoietic malignancies. In this study, we have investigated the role and clinical significance of miR-155 in a Chinese population suffering from GBC and compared the results with nonneoplastic inflammation.

**Methods:**

Tissue specimens were collected on 50 patients of Gall Bladder Carcinoma and 10 patients suffering from nonneoplastic inflammation who have undergone surgeries at the Department of Pathology, Renji Hospital, Shanghai, from January 2019 to January 2020. We performed profiling of miR-155 expression in both nonneoplastic and gall bladder carcinoma tissues by QRT-PCR.

**Results:**

Expression levels of miR-155 were found to be extremely high in GBC patients in comparison to the nonneoplastic tissues (^*∗*^*P* < 0.05), as high miRNA is correlated with TNM stages. Further results noted were that miR-145-5p expressed genes mimic the gene expression of STAT1, a downregulation of IRF7 was noted in the GBC, and an activation of STAT1 was significantly noted in carcinoma cells of the gallbladder. Downregulation of PTPRF was also noted during the expression of miR-145.

**Conclusions:**

As downregulation of IRF7 is linked with low rates of survival, it was found that gall bladder carcinoma patients may face high mortality. The STAT-1 expression of unregulated in GBC patients was also noted.

## 1. Introduction

The most common type of carcinoma in the biliary tract is gall bladder carcinoma (GBC) and is also the third one of most common malignancy conditions of the digestive tract. The most common reason for gallbladder carcinoma is cholesterol gallstones, the condition which leads to chronic inflammation in more than 75% of patients [1, 2].

Ulcerative colitis, chronic *Salmonella typhi*, liver flukes, paratyphoid infections, primary sclerosing cholangitis, and *Helicobacter* infection are amongst the major causes of inflammation, though other factors include exposure to radiations, heavy metals, and pollution and consumption of chemicals. There is a very rare percentage where GBC is linked to hereditary conditions such as neurofibromatosis type, Gardner syndrome, and hereditary nonpolyposis colon cancer [3, 4]. Over 1281 genes are found mutated in GBC. Many studies are available which show that no clear molecular genetic mechanism is available for pathogenesis of gallbladder carcinoma; hence, a detailed research area is available for understanding it, though around 1281 mutated genes were found in people suffering from GBC [5]. Out of the total population diagnosed with gall bladder cancer, around 15–47% can only be treated with surgery whereas most of the patients do not get a chance for surgery as there is early metastasis. Lymph node, adjacent liver metastasis, transperitoneal metastasis, vascular metastasis, and neural metastasis are the factors responsible for gall bladder carcinoma [6–9].

### 1.1. miRNAs

miRNAs are small units of (20–25 nights) single-stranded nonunits which regulate the gene expressions after transcription; thus, the target mRNA gets bound to 3'-UTR 3' untranslated regions. Gene expressions for cell proliferation and differentiation, development, inflammation, apoptosis, and pathological states (autoimmune, cancerous, etc.) are regulated by miRNAs. Due to alteration in expression patterns for cancer and stability in clinical specimens, there is a clear possibility of using miRNA as a biomarker for prognosis and diagnosis of cancer [10–12].

### 1.2. STAT

Signal transducers and activators of transcription is a family of factors of transcription present in the cytoplasm and comprising 7 different members, STAT1, 2, 3, 4, 5A, 5B, and 6 (Darnell Jr., 1997; [13]).

These factors from transcription are activated via a series of extracellular signaling proteins such as growth factors, cytokines, and hormones which specifically attach to cell-surface receptors.

In the current study, 50 GBC patients and 10 nonneoplastic patients were considered for the study. GBC and nonneoplastic tissues were separately connected from the Renji Hospital Pathology Department. Then, RNA sequencing was performed using Bioinformatics analysis; thus, a relationship between the gene expression and the tumor cases was explored.

## 2. Materials and Methods

Patients involved in the study: Formalin-Fixed Paraffin-Embedded (FFPE) tissues from 10 gallbladders (normal) and 50 tissues from gallbladder carcinoma were a part of this research. The samples were collected from the Department of Pathology, Renji Hospital, from January 2019 to January 2020 in accordance with the ethical committee of China.

All the analysis and experimentation were performed as per the relevant guidelines as well as regulations from China, where consent for participation from all participants was undertaken.

The study was performed in due accordance to the Declaration of Helsinki. The subjects have signed the informed consent form prior to the commencement of the study.

A total of **50** patients of gall bladder cancer went through resection surgery in Renji Hospital at the time of diagnosis of GBC, and they did not receive any treatment prior to the process of sample collection.

The cases of gall bladder cancer were confirmed by histopathological analysis with the help of pathologists from Renji Hospital, Shanghai. The nonneoplastic normal tissues of gallbladder were obtained from patients who reported severe inflammation and underwent cholecystectomy for a gallstone disease, and these tissues were used as normal tissues for comparison and reference.

**Cell lines:** Cell Bank of the Chinese Academy of Sciences.

### 2.1. RNA Isolation and qRT-PCR

The Nirvana miRNA kit (Ambion, Austin, TX) was used for extraction of total RNA from gallbladder tissues as mentioned in the standard operating procedure from the manufacturer's protocol. The template for CDNA was further amplified by using real-time PCR with a Premix Dimmer Eraser kit- SYBR (TaKaRa). The PCR reactions in real time were performed by using the ABI7900 system (Applied Biosystems). The expression levels were normalized by U6 as an endogenous control. The values of the samples were determined by duplicating reactions and further normalized by U6 CT values from delta CT (ΔCt = CtmiR-155-CtU6).

### 2.2. Slicing and Preserving of Tissues

The tissues from both gall bladder cancer cases and nonneoplastic normal tissues of gallbladder were embedded in OCT (Tissue-Tek). Then, various tissue sections were cut and obtained using a cryostat (Leica CM 1850).

Cells were kept seeded in 24-welled plates and, hence, incubated for a duration of 24 hours prior to getting stained. Tissue sections were further fixed and preserved for a duration of 1 hour using 4% paraformaldehyde at 4°C. Then, for 1 hour, they were blocked in the blocking solution. Immunotechniques were used for staining the tissue sections, and commercially available antibodies were used in the process.

### 2.3. Immunochemistry (IHC) and Immunofluorescence

In totality, 50 gall bladder cancer samples were stained for fluorescent analysis with BrDU (BioIntron) and GFAP (Sigma-Aldrich) antibodies at 4°C overnight and were counterstained with DAPI (4'-6-diamidino-2-phenylindole) (Sigma, St. Louis, MO, USA; 1 : 30, 000). The immunohistopathological staining was evaluated by two pathologists.

For observing, the samples counterstained with DAPI were also cleared by CUBIC solution. A fluorescent microscope was used (BX51N-34-FL2; Olympus) to capture the images along with a TCS SP8 confocal laser microscope from Leica Microsystems.

The images were captured and analyzed using analysis FIVE software on an Olympus microscope (Olympus, Tokyo, Japan).

A BrDU detection technique was developed as an alternative methodology for precise evaluation of mitogenesis occurrence and stages in the cancer cells of the gallbladder. DAPI staining was performed for gross cell morphology and to determine the number of nuclei.

### 2.4. miRNA Profiling

miRNA profiling was performed on normal tissues (nonneoplastic) and **50** tumor tissues of the gallbladder. The clinical pathological data of all these GBC patients are summarized in Table 1.

### 2.5. Statistical Analysis

The data presented in the study are mean ± SEM. Two-tailed unpaired Student's test and Pearson's Χ2-test have been used to perform the analysis of the variance by using the log-rank test and Kaplan–Meier method for complexity analysis. The hazard regression model has been used in univariate and multivariate analysis; here, *P* < 0.05 is considered as statistically significant. The analysis was performed using the software of SPSS for Windows (SPSS Inc., Chicago, IL).

## 3. Results

The results have been tabulated, and an understanding was reached on the interrelation between the tumor stages, clinicopathological features exhibited (Table 1), gene expression, upregulation, and downregulation of factors based on the immunohistochemistry, immunofluorescence (Figures 1–3), and microarray (Figure 4).

Interpretation: BrDU detection via the antibody technique was used to analyze the levels of mitogenesis in the tissues obtained from GBC and nonneoplastic tissues. In case-I, the mitogenesis was found prominent as compared to case-II. This helps in determining the interpretation that mitogenic stimulation is an essential feature marked in cancer cells. A signal transduction pathway was activated in the human gallbladder cells. Mutagens increase DNA replication.

Interpretation: nuclear staining was performed by DAPI, and blue fluorescence was observed, which helped in the interpretation of the carcinoma cells and inflammation. Protein expression levels were examined in immunofluorescence where the nuclei were counterstained with DAPI.

### 3.1. Interpretation

The immunohistochemistry localization due to GFAP staining is performed to identify the malignancy and giant tumor cells. When GFAP staining is compared with all types of cells, it is found that highly malignant cells, which are undifferentiated, tend to be less developed and less densely positive. Hence, an inverse relationship exists between the degree of malignancy and GFAP. Thus, a low GFAP content is noted in malignant cells in comparison to the normal cells, which is related to the gill filaments disassembly.

## 4. Discussion

microRNA-155 is found to be overexpressed in many hematopoietic malignant and tumor tissues in cases of lung cancer, leukemia, cervical cancer, breast cancer, colorectal cancer, hepatocellular carcinoma (HCC), gastric cancer, pancreatic ductal adenocarcinoma, and renal cell carcinoma (RCC) [14–16].

GBC is commonly diagnosed at advanced stages, mainly due to lack of specific symptoms [17]. Even after major advances in the diagnostic procedures, techniques, and therapeutic management which add to the hope, still the prognosis is poor in gall bladder cancer patients [18].

microRNA-155 (miR-155) expression levels: miR-145-5p expression leads to activation of STAT1 signaling.

In the experimentation when a collective analysis of the IHC was conducted, it was found that the cell proliferation and colonization were significantly reduced. The expression of genes as expressed by miR-145-5p is similar to the signal transducer and activator of transcription 1 (STAT1) pathway which is a majorly tumor suppressor. In the carcinoma cells of gall bladder, the activation of STAT1 was significantly found in comparison to the nonneoplastic carcinoma cells. A downregulation of PTPRF was also noted during the expression of miR-145 which might be involved in the regulation of STAT1 [19]. A downregulation of IRF7 was also found in gall bladder cells, which is linked to low survival rates of gall bladder carcinoma patients.

This study demonstrated the role that mRNA played in the gallbladder carcinoma, which brought light for patients that suffer from disease. However, the limitation is that the concrete mechanism was not clarified. Therefore, further studies are needed to explain the mechanism.

## 5. Conclusions

Hence, it was concluded that the downregulation of PTPRF (protein tyrosine phosphatase receptor type F), activation of STAT-1, and cell proliferation were noted in gallbladder carcinoma cells in comparison to the nonneoplastic cells. The concrete mechanism was not clarified. Therefore, further studies are needed to explain the mechanism.

## Figures and Tables

**Figure 1:** Immunofluorescent images of gall bladder cancer and nonneoplastic tissues for analysis of mitogenesis.

**Figure 2:** Immunofluorescent images of gall bladder cancer and nonneoplastic tissues for analysis of mitogenesis.

**Figure 3:** Immunofluorescent images of gall bladder cancer and nonneoplastic tissues for analysis of malignancy using GFAP.

**Figure 4:** miRNA microarray profiling of nonneoplastic gallbladder tissues and gall bladder carcinoma tissues.

**Table 1:** Correlation between miR-145-5p expression levels and its clinicopathological features.

Characteristic	miR-145-5p expression		miR-145-5p expression		*P* value
	(High, *n* = 27)	%	(Low, *n* = 23)	%	
Age (y)				0.704
<55	12	0.24	9	0.18	
≥55	15	0.3	14	0.28	
Gender					0.826
Male	9	0.18	7	0.14	
Female	18	0.36	16	0.32	
Liver metastasis					0.022
Yes	13	0.26	4	0.08	
No	14	0.28	19	0.38	
TNM stage					0.495
I + II	7	0.14	8	0.16	
III + IV	20	0.4	15	0.30	
Location of the tumor					0.749
Body or bottom	21	0.42	17	0.34	
Neck or duct	6	0.12	6	0.12	

^*∗*^ *P* < 0.05 was considered statistically significant; the *χ*2 test was performed. Higher levels of miR-145-5p were noted in the TNM stages and in liver metastasis.

## Data Availability

The data used to support this study are available from the corresponding author upon request.

## Abbreviations

GBC: Gall bladder cancer
PTPRF: Protein tyrosine phosphatase receptor type F
STAT-1: Signal transducer and activator of transcription 1
miR-155: microRNA-155
HCC: Hepatocellular carcinoma
GFAP: Glial fibrillary acidic protein
DAPI: 4′,6-Diamidino-2-phenylindole
Bride: Bromodeoxyuridine
qRT-PCR: Real-time quantitative reverse transcription PCR
IRF7: Interferon regulatory factor 7
IHC: Immunochemistry.

## References

[1] Kayahara M., Nagakawa T. (2007). Recent trends of gallbladder cancer in Japan. *Cancer*.

[2] Sanders G., Kingsnorth A. N. (2007). Gallstones. *BMJ*.

[3] Shukla H. S. (2006). Gallbladder cancer. *Journal of Surgical Oncology*.

[4] Ishiguro S., Inoue M., Kurahashi N., Iwasaki M., Sasazuki S., Tsugane S. (2007). Risk factors of biliary tract cancer in a large-scale population-based cohort study in Japan (JPHC study); with special focus on cholelithiasis, body mass index, and their effect modification. *Cancer Causes & Control*.

[5] Bartel D. P. (2009). MicroRNAs: target recognition and regulatory functions. *Cell*.

[6] Dutta U. (2012). Gallbladder cancer: can newer insights improve the outcome?. *Journal of Gastroenterology and Hepatology*.

[7] Pilgrim C., Usatoff V., Evans P. M. (2009). A review of the surgical strategies for the management of gallbladder carcinoma based on T stage and growth type of the tumour. *European Journal of Surgical Oncology*.

[8] Tsukada K., Kurosaki I., Uchida K. (1997). Lymph node spread of carcinoma of the gallbladder. *Cancer*.

[9] Misra M. C., Guleria S. (2006). Management of cancer, gallbladder found as a surprise in a resected gallbladder specimen. *Journal of Surgical Oncology*.

[10] Hatfield S., Ruohola-Baker H. (2007). MicroRNA and stem cell function. *Cell and Tissue Research*.

[11] Chen Y., Stallings R. L. (2007). Differential patterns of MicroRNA expression in neuroblastoma are correlated with prognosis, differentiation, and apoptosis. *Cancer Research*.

[12] Uchino K., Ochiya T., Takeshita F. (2013). RNAi therapeutics and applications of MicroRNAs in cancer treatment. *Japanese Journal of Clinical Oncology*.

[13] Lin C. C., Wei J., Ramkrishna M., Feixiong C. (2015). Regulation rewiring analysis reveals mutual regulation between STAT1 and miR-155-5p in tumor immunosurveillance in seven major cancers. *Scientific Reports*.

[14] Han S., Yang S., Cai Z. (2015). Anti-Warburg effect of rosmarinic acid via miR-155 in gastric cancer cells. *Drug Design, Development and Therapy*.

[15] Khalife J., Radomska H. S., Santhanam R. (2015). Pharmacological targeting of miR-155 via the NEDD8-activating enzyme inhibitor MLN4924 (Pevonedistat) in FLT3-ITD acute myeloid leukemia. *Leukemia*.

[16] Erbes T., Hirschfeld M., Rücker G. (2015). Feasibility of urinary microRNA detection in breast cancer patients and its potential as an innovative non-invasive biomarker. *BMC Cancer*.

[17] Kijima H., Wu Y., Yosizawa T. (2014). Pathological characteristics of early to advanced gallbladder carcinoma and extrahepatic cholangiocarcinoma. *Journal of Hepato-Biliary-Pancreatic Sciences*.

[18] Igami T., Ebata T., Yokoyama Y. (2015). Combined extrahepatic bile duct resection for locally advanced gallbladder carcinoma: does it work?. *World Journal of Surgery*.

[19] Darnell J. E. (1997). STATs and gene regulation. *Science*.

